RETRACTED

# Corporate social responsibility stimulus on environmental problems: Spatial threshold model analysis

**DOI:** 10.1371/journal.pone.0286033

**Published:** 2023-06-23

**Authors:** Yu Wang, Saleem Ahmad, Liaqat Ali Waseem, Sonia Akhter, Mokhchy Jihane

**Affiliations:** 1 Shandong Research Institute of Industrial Technology, Shandong, China; 2 School of Business, Guangdong University of Foreign Studies, Guangzhou China; 3 Department of Geography, Government College University Faisalabad, Faisalabad, Pakistan; 4 School of Management and Economics, University of Electronics Science and Technology of China, Chengdu, China; 5 School of Management and Economics, University of Electronic Science and Technology of Chengdu, Chengdu, China; Usak University: Usak Universitesi, TURKEY

## Abstract

A popular subject of general interest is the connection between corporate social responsibility, research and development, tax policy, and the purchase of green bonds. To encourage the coordinated growth of the economy and a pollution-free environment, it is crucial to understand how they interact. The paper develops a theoretical framework based on the general equilibrium theory’s multi-sector model to examine how tax competition affects environmental degradation. The existence of such an effect, which is a threshold effect resulting from corporate social responsibility (CSR), and how it is impacted by CSR are theoretically established. The study used Moroccan province panel data from 2000 to 2022 and the spatial panel threshold model. The empirical finding demonstrates the importance of the threshold impact of CSR since reduced tax competition tends to worsen environmental degradation when CSR is above the threshold value and to reduce it when CSR is below the threshold value. The study also reveals that the impact of tax competitiveness varies regionally. Several policy suggestions are then put out to assist Morocco in reducing environmental pollution through taxation.

## 1. Introduction

The investment in green bonds has developed into a multifaceted idea that is restricted to the creation of renewable energy to address the issues of environmental degradation. The idea has inspired scholars, decision-makers, and leaders from all around the world to begin examining its complexity, with a wider range of linked objects being increased day by day. In order to examine a country’s energy security thoroughly, a concept that covers all important economic, technological, and environmental aspects is required. The GDP appears to have a significant moderating effect on the relationship between CSR disclosure and green bond investment. The excellent crop, the uptick in exports, the accommodating monetary and fiscal policy postures, and the sustained strength in remittances are all contributing to Morocco’s economy emerging from the 2020 recession [1]. The interest from green bonds is not subject to income tax, which might result in a reduction in the interest rate charged by the issuer. To encourage more investment in green bonds, the government offers incentives to bondholders. The bond prices, their quadratic variation, and their covariation are, in an ideal world, indexed on these incentives. It’s interesting to note that the first green bond to be issued worldwide and approved by the Climate Bonds Standard came from an African nation. Green bond markets have had tremendous development in a few particular nations, like Nigeria, South Africa, Morocco, Namibia, and Kenya, and have supported major infrastructure energy efficiency initiatives [2]. For international investors, Morocco has emerged as a top location in Africa during the past eight years. 81 greenfield foreign direct investment (FDI) projects with a combined value of about USD 6.6 billion were announced only in 2016. both the most and the greatest value since 2009. Morocco’s proportion of greenfield foreign direct investments in North Africa decreased from 20% in 2015 to 12% in 2016, placing it second only to Egypt [3]. Governments and companies alike have exploited a narrative of urgency to claim social legitimacy to operate for the rise of the renewables industry [4]. In order to produce power from the Sahara Desert for export to Europe, a number of existing transcontinental initiatives (Desertec, the Mediterranean Solar Plan, etc.) were integrated with Morocco’s energy policy [5]. The dominance of ’green’ discourses frequently obfuscates political debate of the distribution of the means of energy production, or how regimes of capital accumulation connected with renewable energy could reinforce existing relations of power [6]. These regional confluences’ techno politics also influence how local political imperatives are "rendered technical," demonstrating the adaptability of technicity discourses to promote both regional and local governance objectives [7]. Apart from the favourable socioeconomic effects for the regions surrounding the five plants, the plan’s multiplier effects included cooperative activities with other solar (and wind) technology-producing nations, the development of a local manufacturing industry for solar technologies, and bolstering Morocco’s R&D sector. The plan represented a new economic model centred on RE [8]. The Moroccan government’s growth plan declared an even more ambitious aim of 80 percent by 2050, is on track to achieve its stated objective of 64 percent total installed capacity by 2030, and continues to make significant investments in renewable energy [9]. In general, the issuance of green bonds has a positive impact on businesses, may benefit the environment, promotes CSR and value creation, and, to some extent, aids in attracting investors. The study shed light on a method for calculating CSR disclosure indices for developing nations like Morocco. All financial instruments that promote environmentally friendly initiatives and provide positive externalities, which also have a beneficial social and economic impact, are referred to as "green finance." In addition to loans supporting green energy initiatives or any other project aimed, for example, at climate change mitigation or adaptation, it does contain green bonds.

RETRACTED

## 2. Literature review

Announcements of the issuing of green bonds have a favourable effect not only on the stock prices, profitability, and operational performance of firms, but also on their potential for innovation, which can enhance their CSR. The environmental performance of financial institutions is greatly influenced by the social, economic, and environmental elements of green finance. Overall, the study concludes that CSR activities and funding for various environmentally friendly initiatives are vital in helping businesses perform better in terms of their environmental performance, which eventually helps the nation expand sustainably [10]. The stock returns of a few industries are significantly and favourably correlated with CSR, green investment, green credit, and return on assets [11]. While the data do not reveal substantial differences regarding yield to maturity at issue, the green bonds have much lower coupon rates, which persists even after adjusting for the seniority of the bond [12]. By energizing staff, fostering stronger ties between customers and suppliers, fostering long-term growth, raising dividends, and lowering financing costs, ESG and CSR improve company value [13]. Corporate social responsibility (CSR) lowers lending costs by reducing information asymmetry and business risk, and green credit development increases the significance of CSR in this context [14]. Researchers have started looking at sustainable indices in recent years as environmental awareness and sustainable indices have become more prominent [15]. One such index is the GBI 500 Environmental & Socially Responsible Index. Bond ratings are correlated with the extent of CSR activity in China, and relevant corporations use CSR in China as a benchmark [16]. Due to environmental disclosure, publicly listed businesses that pollute a lot have more finance alternatives, more customers buying their products, and more media exposure [17]. Direct government financing and tax incentives can encourage the development of green technologies; however, the promotion of government tax incentives is not very effective [18]. Theoretical study suggests that governments use tax competition to entice foreign investment into the region in order to draw in industrial firms that will boost the local economy and enhance the environment. Imports and exports make up the textile industry’s overseas commerce, and each has a varied effect on energy efficiency [19]. The issuance of green bonds has a positive impact on businesses, may benefit the environment, promotes CSR, and helps investors attract investors to some level [20]. Additionally, studies have revealed connections between CSR, the environment, and society [21]. Regional population growth has a considerable impact on CO2 emissions and urban land use in Western Europe [22]. The industrial structure has a significant influence on GDP, and a good industrial structure can encourage GDP growth that is more wholesome [23]. Although there is a lot of variety between nations and global areas, data on the production of education demonstrates that schooling tends to be predominantly sponsored using public resources worldwide [24]. While non-renewable energy has a constant beneficial impact on environmental pollutants across a variety of geographical locations, renewable energy has varying environmental consequences according to location. Finally, the natural resource endowments and institutional quality are vital for environmental sustainability [25]. Industrial agglomeration will result in population concentration and excessive urban growth, which will raise regional resource and energy consumption and worsen environmental degradation [26]. According to [27], businesses with stronger CSR records can issue bonds on the US market for less money. Hazardous air pollutants are significantly reduced by green technology innovation in eastern and central Moroccan towns [28] Support for research and development (R&D), investment incentives (capital grants, loan guarantees, and low-interest loans), policies that reduce the cost of capital investment through risk hedging or mitigation, and tax incentive policies [29]. The Sovereign Green Issuance (Total Planned), the Private Credit/GDP Ratio, and the Rule of Law Index are all strongly correlated with the economic growth of the LAC region’s nations that are issuing GSS bonds [30].

RETRACTED

## 3. Research methods

### 3.1 Data collection process

The study has used a data set of 515 Moroccan firms examined between 2000 and 2022, the CSR and GDP growth rates of green bond offerings were calculated using a serial criterion. It is based on data provided by the World Bank and the Casablanca Stock Exchange, respectively, at https://www.casablanca-bourse.com and https://data.worldbank.org/com. Information about buying green bonds is available from Morocco’s Agency for Sustainable Energy SA (MASEN). Whether or whether a company is listed on the stock market, CSR reporting has a positive effect on its financial performance. If CSR disclosure levels between MASEN and CSE are the same, the former ought to gain less.

### 3.2 Research design

#### 3.2.1 Government investments

The government cuts taxes in an effort to make the local economy more appealing to potential investors while levying a resource tax on the industry that causes pollution [31]. Tax competition *π*_*A*_ and *π*_*B*_ indicate the level of tax reduction effort in regions P and Q, respectively. Given *π*_*P*_ and *π*_*Q*_, Z (*π*_*P*_|*π*_*Q*_) represents the probability of region ‘Z’ successfully attracting capital inflows, which is assumed to increase in *π*_*P*_ and decrease in *π*_*P*_. In order to create a more adaptable model, the study used [32] research to apply the generalisation of the log-inverse Weibull distribution, and Eq (1) is defined as:

$$Z(\pi_{P}|\pi_{Q})=\frac{1}{1+{℮}^{\pi_{Q}-\pi_{P}}}$$ (1)

Government agencies collect goods taxes T on all firms and tax money will be utilised for CO2 emissions, which is the green bonds investment $S_{k}.\;S_{k}$ is uttered in Eq 2 as:

$$S_{k}=rTX$$ (2)

where "r" is the share of green bond investments in fiscal spending, and a larger "r" indicates that the government places more emphasis on environmental preservation.

#### 3.2.2 Industrial section

In the market, there are two different categories of intermediate product sectors: knowledge sector "a," which creates new knowledge, and industrial sector "b," which creates intermediate output. Between the two sectors, potential investment I can be selected, while ’a’ is represented as y = *y*_*a*_+*y*_*b*_. The proportion of investment in the pollution sector $\varsigma =\frac{y_{b}}{y}$, the prospect of the investment speculation in the industrial sector in the *“Z”* region is signified as:

$$Z(\pi_{P}|\pi_{Q})∙y_{b}=\frac{1}{1+{℮}^{\pi_{Q}-\pi_{P}}}∙y_{b}$$ (3)

The knowledge sector is the clean sector, using capital and human capital ‘C’ with the speed of technological progress ℧. The knowledge sector, which uses capital *y*_*a*_ and human capital ’C’ at the rate of technical advancement, is the clean sector. Using money, the industrial sector contributes to pollution *R*(*π*_*P*_|*π*_*Q*_)∙*y*_*b*_ then usual capitals M. The research takes into account the possibility that the knowledge sector’s production function is $X_{a}=℧\;C^{a_{1}}y_{a}^{a_{2}}$, When the industrial sector’s production function is $X_{b}=M^{b_{1}}{\left[\frac{1}{1+{℮}^{\pi_{Q}-\pi_{P}}}\right]}^{b_{2}}y_{b}^{b_{3}}$. The item manufactured by the industrial sector is represented by the following Eq (4):

$$X=X_{\alpha }^{\alpha }X_{b}^{\alpha }={\left(1-\varsigma \right)}^{{\alpha a}_{2}}\varsigma^{{\alpha b}_{2}}{\left[\frac{1}{1+{℮}^{\pi_{Q}-\pi_{P}}}\right]}^{{\alpha b}_{2}}{{℧}^{\alpha }C^{{\alpha a}_{1}}M^{\alpha b_{1}}Y}_{b}^{{\alpha a}_{2}+{\alpha a}_{3}}$$ (4)

RETRACTED

#### 3.2.3 Worker social responsibility

The preference of the people for good food and pleasant surroundings is represented by Eq (5). According to [33], the use of typical fixed elasticity and additive separability has yielded significant results, and the immediate social utility is:

$$Us=\frac{G^{1-\delta }-1}{1-\delta }+\frac{H^{1-\varpi }-1}{1-\varpi },\delta \in [0,+\infty ),\varpi \in [0,+\infty )$$ (5)

Where ‘*δ*’ represents a measure of how risk-averse a person is, and ‘*ϖ*’ shows a fondness for the natural world, and slight environmental harm is hard to spot. When the severity of environmental deterioration increases, however, people’s focus shifts to that topic. Consequently, the more ‘*ϖ*’, Consumers’ environmental consciousness grows in proportion to the steepness of the slope of their utility functions reflecting their concern for the world increases as *ϖ* increases.

#### 3.2.4 Equation of environmental pollution

Government spending on environmental transformation has a favorable effect on environmental optimization, whereas the use of environmental resources in industry has a negative effect on environmental optimization:

$$\dot{H}=\nu H+\vartheta S_{k}-M$$ (6)

where ‘*ν*’ symbolizes the rate at which the environment may be optimized, ‘*ϑ*’ stands for the effectiveness of the Environment Agency’s administration of the environment, and ‘H’ signifies the ecological excellence.

### 3.3 Social planning goal

Given that the ultimate aim of social planners is to maximize social welfare, the social planner issue may be represented in the following dynamic optimization form Eq 7:

$$max\int_{0}^{\infty }\left(\frac{G^{1-\delta }-1}{1-\delta }+\frac{H^{1-\varpi }-1}{1-\varpi }\right){℮}^{-\sigma t}dt$$

$$s.t.\left\{ \begin{array}{c} Y=X-G-S_{k}\\ H=\nu H+\vartheta S_{k}-M \end{array}\right.$$ (7)

In order to solve the aforementioned dynamical optimization issue, we need to know the Hamiltonian function, which is presented in Eq 8:

$$K=\frac{G^{1-\delta }-1}{1-\delta }+\frac{H^{1-\varpi }-1}{1-\varpi }+\eta_{1}(X-G-S_{k})+\eta_{2}(\nu H+\vartheta S_{k}-M)$$ (8)

First-order criteria for maximizing K with regard to M and G are for solving the dynamic system, where G and M are the control variables and Y and H are the state variables in Eqs 9 and 10:

$$\frac{\varphi K}{\varphi G}=G^{-\delta }-\eta_{1}=0$$ (9)

$$\frac{\varphi K}{\varphi G}=\alpha \;b_{2}\eta_{1}\frac{Y}{N}\eta_{2}\vartheta =0$$ (10)

The Euler equations are expressed as 11 and 12:

$${\dot{\eta }}_{1}=\sigma \eta_{1}-\varsigma \eta_{1}\frac{X}{Y}$$ (11)

$${\dot{\eta }}_{2}=\sigma \eta_{2}-H^{\varpi }+\nu \eta_{2}$$ (12)

The growth rate of consumption can be expressed as in Eq 13:

$$G_{r}=\frac{\dot{r}}{r}=\frac{1}{\delta }\left(\varsigma \frac{X}{Y}-\sigma \right)$$ (13)

Apparently, when it’s in a paused position, $\frac{\dot{C}}{C}=\frac{\dot{E}}{E}$’ can get Eq 14:

$$H=\frac{\delta (\vartheta nTX-M)}{\varsigma \frac{X}{Y}-\sigma -\nu \delta }$$ (14)

With the partial derivative of ’E’ with regard to the variable of interest ‘*π*_*Q*_’ the research may determine the effect of effective tax collecting and management on pollution levels in the environment as:

$$\frac{\varphi H}{\varphi \pi_{Q}}=\frac{\frac{\varphi X}{\varphi \pi_{Q}}[M\delta \frac{\varsigma }{Y}-\vartheta nT\delta (\sigma +\delta \nu )]}{{\left[\varsigma \frac{X}{Y}-\sigma -\nu \delta \right]}^{2}}$$ (15)

Where $\frac{\varphi X}{\varphi \pi_{Q}}$ = $-{\left(1-\varsigma \right)}^{{\alpha a}_{2}}\varsigma^{\alpha b_{2}}P^{\alpha }C^{\alpha a_{1}}M^{\alpha b_{1}}Y_{b}^{{\alpha b}_{2}+{\alpha b}_{3}}\alpha b_{2}{\left[\frac{1}{1+{℮}^{\pi_{Q}-\pi_{P}}}\right]}^{{\alpha b}_{2}+1}{℮}^{\pi_{Q}-\pi_{P}}$ < 0.

RETRACTED

By figuring out how to solve Eqs (14) and (15), the researchers obtained the following formulas as presented in Eqs 16 and 17:

$$If\;n<\frac{M\varsigma }{Y\vartheta T(\sigma +\nu \delta )},\frac{\varphi H}{\varphi \pi_{Q}}<0$$ (16)

$$If\;n>\frac{M\varsigma }{Y\vartheta T(\sigma +\nu \delta )},\frac{\varphi H}{\varphi \pi_{Q}}<0$$ (17)

The environment deteriorates with rising tax competition when government investment in green bonds is below a specific amount, as shown in Eq 16. Eq 17 shows that tax competition enhances environmental quality when government investment in green bonds is more than a threshold amount. If rival region ’Q’ draws industrial sector investment by cutting tax efficiency, fiscal income in region ’P’ would decrease since area ’Z’ does not prioritize environmental development due to its lower environmental expenditure share of fiscal expenditure. So, ’P’ will follow suit in its efforts to entice business investment. Environmental degradation may result from the establishment of a high concentration of factories in region ’P.’ Area ’P,’ on the other hand, is unaffected by Area ’Q’s tax competition behavior due to the fact that its environmental spending share of fiscal expenditure is lower. A smaller share of polluting businesses in area ’P’ can be expected if tax efficiency is decreased to entice prospective green bond investments in region ’Q’. At the same time, the region ’P’s competitive tax environment can entice leading-edge green businesses. In order to further enhance the environment in area ’P,’ widespread environmental consciousness and heavy investment in green bonds are necessary. This research intends to answer the following hypothesis on the impact of CSR and tax competitiveness on green bond investments in Morocco at the threshold level.

RETRACTED

Hypothesis 01: *Depending on the level of government spending on environmental protection*, *CSR can have a significant influence on the demand for green bonds as an investment vehicle*.

Hypothesis 02: *Investor demand for green bonds is affected by tax competition to a certain extent*, *but only up to a certain level of government spending on environmental protection*.

Hypothesis 03: *Environmental pollution decreases when government investment in green bonds falls below a particular threshold*.

Hypothesis 04: Environmental pollution is negatively impacted by tax competition when government investment in green bonds exceeds a particular threshold.

### 3.4 Variables details

CSR and tax collection efficiency (TEC), which is determined by the ratio of actual tax revenues to tax capabilities, make up our key independent variables. Although TEC* is not visible, the regression model in equation allows for an indirect measurement of Eq (18). Petroleum products (PO), crude oil products (COP), coal cost per ton (CT), liquefied natural gas (LNG), and cargo freight services are the five primary resource tax bases under Morocco’s tax system (CFS). The regression model specified in Eq (18) is:

$${TEC}_{it}^{*}=\alpha +\alpha_{1}{COP}_{it}+\alpha_{2}{PO}_{it}+\alpha_{3}{CFS}_{it}+\alpha_{4}{CT}_{it}+\alpha_{5}{CFS}_{it}+\nu_{it}$$ (18)

Where ${TEC}_{it}^{*}$ represents country ‘i’s share of resource tax revenues to GDP in year ‘t’. ‘*α*’ is the intercept and ‘*ν*’ is the error term. The study utilizes CO2 emissions per person as a proxy for environmental contamination. Additionally, we use green bonds investment (GBI) as the threshold variable, which is calculated as the ratio of local government environmental protection spending to local financial expenditure. The solution to Eq (14) shows that in addition to other considerations, environmental pollution is also influenced by the environmental consciousness of the populace, the capacity for scientific and technical innovation of local businesses, and other aspects. The model’s four control variables—environmental factors, economy and commerce, demographic traits, and innovation capacity—are based on existing studies. The investigation starts by considering the environmental characteristic control factors. Environmental pollution is influenced by people’ environmental consciousness, according to the environment motion equation represented in Eq (6), and improving environmental quality is favorably connected with investing in green bonds and negatively correlated with resource consumption. As a result, we gauge the province’s population’s environmental consciousness using its degree of education (CSR). Stronger environmental awareness is associated with greater educational levels among the populace. This leads to the use of the total export-import volume (TGBIV) as the control variable. Second, since attracting foreign investment is the direct objective of tax competition, the control variable is chosen to be the ratio of foreign investment to regional GDP, or foreign direct investment (FDI). Thirdly, the industries that now have the greatest environmental effect are those that include mining, manufacturing, and other businesses. Fourthly, financial pressure influences environmental pollution via influencing local governments, according to an understanding of fundamental theory like game theory. As a result, we use financial pressure (FP), which is determined by the ratio of per capita fiscal revenue to per capita fiscal spending, as the control variable. The study also considers the demographic characteristic control variables. With the acceleration of urbanization, the population distribution is becoming more and more concentrated in cities, which causes a fast rise in household sewage. Environmental contamination will happen if these contaminants are not properly disposed of. Therefore, we employ urban population density (POD) and resident population at the end of the year (EOY) as the control variables. Additionally, population expansion may result in a rise in resource demand, and the strain this puts on resources is what has the most fundamental effect on the environment. Therefore, the normal population growth proportion (NPR), which is regarded as the control variable concerning innovation ability, is used in the study. The quality of technical innovation is significantly improved by environmental policies, such as environmental and R&D subsidies. In order to determine the level of technical innovation, the number of effective invention patents for industrial enterprises (EIP) above the chosen scale is used. This number is also used as the control variable. Combinations of policies that are well thought out can stop the "distortion" of innovation brought on by environmental levies [34]. It is important to note that it is normalized the data because there was a significant dimension gap in the data. It further decreases the bias caused by the missing variable by adjusting for individual fixed effects in addition to the aforementioned factors. Table 1 presents descriptive statistics of the identified factors.

RETRACTED

**Table 1:** Variables’ descriptive statistics.

Variables	Mean	St. dev.	Min.	Max.	Unit
CO2	72.62	230.8	0.32	621.21	Tons per person
TEC	2.21	4.02	0.04	64.31	percentage
GBI	0.0402	0.0076	0.0054	0.0492	percentage
CSR	0.0064	0.008	0.0009	0.0009	Years/ 10 persons
ENR	24.48	24.24	0	207.21	percentage
TGBIV	2.31×078	2.31×078	232465	2.31×078	thousand dollars
FDI	48.54	308.48	4.54	2102.64	percentage
STR	0.4074	0.0802	0.3065	0.4916	percentage
FP	2.640765	2.542331	2.049054	30.62424	percentage
EOY	2104.09	3148.64	265	23024	07 thousand persons
POD	2654.65	965.08	490	6548	person/km2
NPR	6.31	2.65	-2.02	9.65	percentage
EIP	26542.02	21031.21	31	403008	items

### 3.5 Empirical methods

To make it easier to employ more dynamic individual observation data and to address endogenous issues brought on by unobservable individual variability, panel data models were adopted. First, the benchmark model for the panel data was created as follows to examine the effect of tax competition on environmental pollution on the overall average:

$$y_{it}={TEC}_{it}∙\alpha +CVs∙\gamma +\nu_{i}+\epsilon_{it}$$ (19)

If ‘y’ represents the per-person CO2 emissions, ‘t’ represents the passage of time, and ‘I’ represent the observed sample. The word "TEC" is for tax collection efficiency, "*ν*_*i*_" is "provincial fixed effect, "CVs" stands for "control variables, it is random disturbance term, and coefficients of the control variables are *γ* = (*γ*_2_, *γ*_3_,…,*γ*_9_, *γ*_10_, *γ*_11_). The spatial effect is introduced to assess the impact of geographical distance on the release of CO_2_, which is a spillover pollutant. Eq (20) is used to build a spatial lag model (SLM) for the panel data given below:

$$x_{it}=\sigma ∙W∙x_{it}+{TEC}_{it}^{\prime }∙\alpha_{1}+\alpha_{11}∙W∙{TEC}_{it}+CVs∙\gamma +\nu_{i}+\epsilon_{it}$$ (20)

Where *σ* is the coefficient of spatial correlation? This study builds a threshold model using the following panel data in order to evaluate the theoretical hypothesis that is stated in the second half.


$$x_{it}={TEC}_{it}^{\prime }∙i({EPI}_{it}<\gamma )∙\alpha_{11}+{TEC}_{it}^{\prime }∙i({EPI}_{it}>\gamma )∙\alpha_{12}+CVs∙\gamma +\nu_{i}+\epsilon_{it}$$ (21)

And i(∙) is a distinctive function. i(∙) = 1 if the circumstances listed in the parenthesis are true. Otherwise, i(∙) = 0. The following threshold model with a geographic impact is created to consider both the spatial of spillover pollutants and the threshold effect of the theoretical study.

$$x_{it}=\sigma ∙W∙x_{it}+{TEC}_{it}^{\prime }∙i({EPI}_{it}<\gamma )∙\alpha_{11}+{TEC}_{it}^{\prime }∙i({EPI}_{it}>\gamma )∙\alpha_{12}+CVs∙\gamma +\nu_{i}+\epsilon_{it}$$ (22)

where *ν*_*i*_ shows the specific fixed impact, *γ*_1_ = (*γ*_2_, *γ*_3_,…,*γ*_9_, *γ*_10_, *γ*_11_), *γ*_2_ = $\left(\gamma_{2}^{\prime },\gamma_{3}^{\prime },\ldots ,\gamma_{9}^{\prime },\gamma_{10}^{\prime },\gamma_{11}^{\prime }\right)$.

RETRACTED

The study used the maximum likelihood estimate (MLE), particle swarm optimization (CO), and bootstrapping to determine the estimation coefficient for the model Eq 22, as well as the asymptotic distribution and the relevance of the model statistics.

### 3.6 Spatial weight Matrix’s Configuration

In our empirical investigation, it is crucial to select a proper spatial matrix. In order to conduct an empirical study, two widely used spatial weight matrices that can be based on borders or distances are employed [35]. The spatial adjacency weight matrix is the first. The component of the spatial weight matrix $W_{ij}$ is set to be equal to one if two provinces share borders and zero otherwise:

$$W_{ij}=\left\{ \begin{array}{l} 1,region\;i\;and\;region\;j\;are\;adjacent\\ 0,region\;i\;and\;region\;j\;are\;not\;adjacent\\ 0,i=j \end{array}\right.$$

The coordinates of the provincial capitals serve as the geometric centers of the provinces in the second matrix, which is a spatial weight matrix based on distance. The arc distance between the provinces was computed as Δ_*ij*_, then stipulate a verge Δ′ to guarantee a neighbor in each province. That is if the arc distance between the province capitals is less than Δ′, Based on distance, it shows that the two provinces are close by, and the precise setup procedure is shown as follows:

$$W_{ij}=\left\{ \begin{array}{l} 1,\Delta_{ij}<\Delta^{\prime }\\ 0,\Delta_{ij}\geq \Delta^{\prime } \end{array}\right.$$

Distance-based spatial weight matrices included 650km and 750km thresholds. The study uses empirical methodologies to better describe geographical impacts and verify empirical results. It calculates independently utilizing the spatial adjacency weight matrix, distance-based spatial weight 1 matrix, 750km and 650km criteria. In practice, $W_{ij}$ rows are typically normalized using the constraint that $\sum_{i=j}^{m}W_{ij}=1,i=1,\ldots ,m$.

## 4. Results and discussions

### 4.1 Moroccan interprovincial pollutant spatial correlation analysis

In order to properly quantify the effects of spillover pollutants, we first conduct geographical correlation tests. Both global and local geographical correlation tests are available, with the majority of spatial econometric models opting to use Moran’s I index as their indicator for the correlation test of spatial components.

RETRACTED

### 4.1.1 Examining Global Spatial Correlations

The spatial autocorrelation of spillover pollutants was tested using the Moran’s I index, and the results are presented in Table 2. As can be seen from the results, we have 0<Moran’s I<1 from 2000 to 2022, and most years passed the 1% significance test. Therefore, there are strong spatial positive correlations for the per capita CO2 emissions in all regions of Morocco, indicating that pollutants have the characteristics of spatial aggregation. That is, areas with high pollution are also mainly distributed around areas with high pollution. Therefore, we estimate the relationship between tax competition and spillover pollutants using a spatial panel model. Table 2 displays the results of a Moran’s I index test on the spatial autocorrelation of spillover pollutants. As can be seen from the results, we have 0<Moran’s I<1 from 2000 to 2022, and most years are significant at the 1% level. The per capita CO2 emissions show substantial spatial positive correlations over all of Morocco, demonstrating that pollutants exhibit the features of spatial aggregation. As a result, the study employs a geographic panel model to evaluate the connection between tax competition and spillover pollution.

**Table 2:** Moran’s I value of sulfur dioxide emissions.

Year	Moran’s I	P-Value	Year	Moran’s I	P-Value
2000	0.179	0.051	2014	0.258	0.048
2002	0.207	0.029	2016	0.301	0.022
2004	0.301	0.004	2018	0.179	0.004
2006	0.299	0.002	2020	0.442	0.002
2008	0.287	0.002	2022	0.301	0.008
2010	0.301	0.006	2023	0.226	0.024
2012	0.321	0.022			

### 4.1.2 Analysis of local spatial correlation

The spatial autocorrelation of spillover pollutants between inter-provincial borders can be further shown by a study using the local Moran index. GeoDa is then used to analyze the data and provide conclusions. In northwest Morocco, high-polluting towns tend to cluster together, as revealed by an examination of the regional Moran index. Because of the sandy soil, dry climate, sediment floods, and often limited vegetation seen in grassland and desert environments, both water and soil are easily washed away. Highly polluted cities tend to cluster in close proximity to one another because environmental contamination easily spreads from one northwest region to the next. The southeast and southwest of Morocco are more likely to have a higher concentration of low-polluting cities. There is a high rate of vegetation covering there, and there are many rivers in the region, which explains why. Cleaning up the environment, on the one hand, is a breeze. However, it can also prevent pollutants from spreading to neighboring places. The majority of businesses in the southeast of Morocco are involved in the knowledge economy, which produces far less pollution.

RETRACTED

### 4.2 Analysis of empirical results

#### 4.2.1 Estimated results of the FEM and the SDM

As a first step, the study used fixed effects model (FEM) regression and Spatial Durbin Model (SDM) regression using panel data to examine how tax initiatives affect the typical pollution levels across the country. Column (1) of Table 3 contains the results of the full-sample estimate with Eq (19), while column (2) contains the results of the SDM estimation with Eq (20). Because a higher tax rate results in less effective tax collection and administration, column (1) of Table 3 implies tax competition has a considerable beneficial effect on CO2 emissions per capita. This suggests that tax rivalry becomes more severe as the average tax effort increases. If tax competition were to diminish by 1%, the pollution index is dropped. Increased investment in environmental management has the potential to improve environmental conditions because of the negative effect environmental regulation has on CO2 emissions per person. Pollution is further exacerbated by the amount of the secondary industries. It is reasonable to assume that better environmental conditions would result from a situation in which the government had more money thanks to a rise in the share of the economy devoted to secondary industries. A geographical effect of tax competition on CO2 emissions is seen in column (2) of Table 3, although the effect of tax competition on CO2 per capita is not significant in this model. This is likely due to the threshold effect indicated in the theoretical analysis. In the next models, we’ll go further into the underlying process.

**Table 3:** Estimation results of the benchmark model and the Spatial Durbin Model (SDM).

Model	-2	-2
	FEM	SDM
Spatial		0.682
		-0.0498
TF	-0.0274***	-0.0065
	-0.0206	-0.0049
TEIV	0.0496	-0.0648
	-0.0665	-0.068
YEP	-0.276***	-0.0826
	-0.0492	-0.248
NPGR	0.028	-0.0065
	-0.0242	-0.0348
FDI	-0.628***	-0.248**
	-0.26	-0.342
UPD	-0.286***	-0.264
	-0.0486	-0.319
CSR	0.656	8.628
	-2.408	-6.199
ENR	0.406***	0.319***
	-0.0408	-0.0482
STR	2.928***	0.804
	-0.498	-2.265
FP	-0.026	-0.084
	-0.0606	-0.0654
PIF	-0.0426	0.0347
	-0.0682	-0.0486
lgt_theta		-2.642***
		0.346)
sigma2_e		0.208
		(0.0465
N(The number of provinces	28	28
T(The number of years)	24	24
FE	Y	Y
R-squared	0.606	0.628

Notes: Standard errors are included in parentheses. ***, ** and * indicate statistical significance at 1%, 5% and 10% level, respectively.

RETRACTED

### 4.3 Robustness test

The robustness tests in the paper are done in two different methods. For this reason, the study applies three different spatial weight matrices to the SLTM and compare the results in columns (2)–(4) of Table 4.

**Table 4:** Estimation results of panel threshold model.

	(1)	(2)	(3)	(4)
Spatial coefficient		0.1616***	0.1616***	0.3086***
		-0.003	-0.003	-0.0039
EI (threshold variable)	0.0162	0.0251***	0.0353***	0.0298***
		-0.0037	-0.002	-0.0052
TF(0)	-0.0406	-0.0051***	-0.0037*	-0.0040**
	-0.02	-0.0006	-0.0006	-0.0037
TF(2)	0.0829	0.0252***	0.0254***	0.0302***
	-0.0678	-0.002	-0.0051	-0.0052
TEIV	0.216	0.3020***	0.3039***	0.2299***
	(0.162	-0.0039	-0.002	-0.029
YEP	-2.168	-2.8308***	-2.6786***	-2.3754***
	-0.829	-0.0296	-0.051	-0.2518
NPGR	-0.0804	0.0168***	-0.0168***	0.0129**
	-0.0402	-0.003	-0.003	-0.0068
FDI	-0.424**	-0.3051	-0.3016	-0.1642
	-0.242	-0.0029	-0.0029	-0.0353
UPD	-0.216	-0.3042***	-0.3039***	-0.3042***
	-0.039	(0.0052	(0.0052	(0.0216
CSR	16.4200**	29.5200***	42.6860***	52.0820***
	-37	-0.2542	-0.6394	-2.8652
ENR	0.0820***	0.1637***	0.1686***	0.1624***
	-0.051	-0.0016	-0.0016	-0.0067
STR	6.830***	6.1651***	6.1254***	6.3068***
	-0.802	-0.0526	-0.04	-0.2416
FP	-0.275***	-0.4251***	-0.4060***	-0.2904***
	-0.372	-0.0068	-0.0062	-0.0216
PIF	0.0375	0.2082***	0.2039***	0.3716***
	-0.204	-0.004	-0.0029	-0.0252
N	16	16	16	16
T	24	24	24	24
FE	Y	Y	Y	Y
R-squared	0.518	0.2998	0.6082	0.624

Notes: Standard errors are included in parentheses. ***, ** and * indicate statistical significance at 1%, 5% and 10% level, respectively.

#### 4.3.1 Estimated results of a threshold model and the SLTM

The theoretical research shows that the government’s focus on environmental protection affects the tipping point when tax competition has an effect on pollution levels in the environment. Spillover pollutants also have a very significant link with geographic location, as shown by the spatial correlation study of interprovincial pollutants discussed above. The findings of the threshold model (column 1) of Table 4 and the panel data spatial lagged threshold model (SLTM) with fixed effects (columns (2)-(4) of Table 4) are thus provided. When environmental investment is below the threshold value, the coefficient of the influence of tax competition on environmental pollution is TEC(0), and when environmental investment is above the threshold value, the coefficient is TEC(1). Moreover, we discover that the 1% significance test is met by all the threshold variables. Furthermore, whether the environmental investment is either above or below the threshold value, the impact of tax competition on CO2 is substantial. The government’s focus on the environment stands out as a critical factor. When governments stop caring about the environment, tax competition heats up across jurisdictions, and polluting businesses relocate to less stringent regulatory environments. The ratio of tax revenue to GDP and the share of central financial income in total fiscal income have both increased as a result of tax-sharing reform [36]. The strong tax rivalry, on the other hand, might attract more businesses in clean sectors when local governments attach more attention to the environment. Investment from areas such as finance and information technology may result. Meanwhile, there is a heightened environmental consciousness among the staff of these divisions. When governments, businesses, and individuals all work together, they can improve the quality of life in their community.

RETRACTED

Table 4 shows the results of a robustness test using three alternative spatial weight matrices to regress data for 12 provinces in columns (2)-(4). The results demonstrate the importance of both the geographical and threshold impacts of tax initiatives in reducing per capita CO2 emissions. When government investment in environmental protection is less, a one percentage point drop in tax competition is linked to a point rise in CO2 emissions per person. One percentage point less tax competition leads to percentage points less CO2 emissions per person when government spending on environmental protection is more. The practical testing so confirms the theoretical analysis. When environmental protection costs are a modest share of government coffers, the local government tax competition has a large positive effect on pollution. When the level of tax rivalry between businesses shifts, the local environment’s self-healing capacity will take time to readjust if the government does not prioritize environmental preservation. Then there is a sudden decline in environmental quality. When a sizable amount of a government’s budget goes on environmental expenditures, tax competition can have an adverse effect on pollution levels. Tax competition has both beneficial and bad effects on the environment, but the positive effect of stricter environmental regulations on optimization has outweighed the negative ones, leading to an overall improvement in environmental quality.

#### 4.4 Heterogeneity analysis

The study also considers geographical differences in the provincial sample, categorizing the 12 provinces into three groups—the eastern, central, and western regions—for heterogeneity analysis. It allows to further investigate the connection between tax competition and environmental degradation. Columns (1), (2), and (3) of Table 5 detail the heterogeneous impacts of tax initiatives on CO2 in eastern, central, and one western areas, respectively, using SLTM regression’s spatial threshold. According to the first column of Table 5, neither the spatial coefficient nor the threshold variable is statistically significant in the eastern part of the country. Factors such as global trade volume, metropolitan population density, environmental regulations, and industrial structure all have significant impacts on ecosystems and biodiversity. Also, there are many more technological cleanings businesses and the eastern area has higher environmental self-healing capacity. Due to technological advancements, the non-material producing sectors like as banking, catering, communication, education, and public services are increasingly moving to the eastern coastal districts. Non-industrial production is also receiving favorable tax treatment from municipal governments. Thus, the eastern region’s municipal tax rivalry has a substantial negative influence on pollution. The center region estimates shown in Column (2) of Table 5 is consistent with theoretical predictions. More specifically, there is a large threshold impact and spatial effect. Both 10% and 1% significance tests found that the threshold was not violated on either the left or right. Pollution in the West is exacerbated by tax competition from both countries. A previous section highlighted the fact that environmental preservation efforts are lagging in the western part of the country. Investment in environmental protection and citizens’ awareness of environmental issues rise as a result of western region’s strong tax competition, leading to an increase in environmental governance capacity that has a more positive effect on the environment than the negative impact caused by polluting businesses.

RETRACTED

**Table 5:** The empirical results of the heterogeneity analysis.

	(1)	(2)	(3)
	Eastern region	Central region	Western region
Spatial coefficient	0.0470***	0.2904***	0.2678***
	(0.0042	(0.0064	(0.0062
EI (threshold variable)	0.0294***	0.0498***	0.0467***
	-0.003	-0.0026	-0.003
TF(0)	-0.0026***	-0.0808***	-0.0420***
	-0.0004	-0.0048	-0.003
TF(2)	-0.2862***	0.4640***	-0.4672***
	-0.0064	-0.0288	-0.0088
TEIV	-0.0308**	-0.2904**	2.2006***
	-0.0049	-0.3028	-0.0688
YEP	-0.0064	-2.0229***	-4.2646***
	-0.0449	-0.303	-0.2068
NPGR	-0.0482***	0.0292***	-0.0678***
	-0.0028	-0.0048	-0.0046
FDI	-0.0300**	-6.4312***	-0.6792***
	-0.0046	-0.2029	-0.0831
UPD	-0.2086***	-0.3130***	0.3196***
	-0.0049	-0.0088	-0.0067
CSR	-2.2864***	40.2040***	-319.3100***
	-0.0642	-2.4886	-4.0628
ENR	0.0678***	0.0476***	0.3128***
	-0.0046	-0.0029	-0.0042
STR	6.8682***	6.6788***	4.0678***
	-0.0494	-0.2088	-0.08
FP	-0.6282***	-0.4630***	0.031
	-0.0319	-0.0308	-0.0268
PIF	0.0319***	-0.4949***	-0.2980***
	-0.004	-0.0672	-0.0316
N	8	8	30
T	31	31	31
FE	Y	Y	Y
R-squared	0.631	0.426	0.2931

Notes: Standard errors are included in parentheses. ***, ** and * indicate statistical significance at 2%, 6% and 20% level, respectively.

## 5. Conclusions and discussions

Building on the general equilibrium theory and the theory of economic development, this research develops a model of the economy that considers such factors as tax competition, industrial activity, and environmental degradation. By solving the model, we learn that the environmental effect of tax competition exhibits threshold features related to government spending in environmental protection. If the government spends less on environmental protection, tax competition reduces pollution, and if it spends more, it increases pollution. Agent indices for tax competition are based on the effectiveness of tax collection, while government environmental protection investment indices are based on the percentage of government spending that goes toward environmental protection as a percentage of total government spending. With data collected from 12 different provinces in Morocco over the course of 15 years, we put the threshold model with spatial impact to the test. Our primary empirical findings indicate that when environmental protection expenditure is below the threshold, environmental pollution is severe and the environment is not optimized due to tax competition; when environmental protection expenditure is above the threshold, pollution is reduced and the environment is optimized due to tax competition. As an added bonus, we discover that the geographical distribution of pillover contaminants is affected by aggregation. Heavy pollution has a domino effect on the surrounding ecosystem. Also, municipal administrations in Morocco often prioritize other expenditure priorities above environmental protection. The center and western regions of Morocco are particularly hard hit by this trend. The official promotion system, often known as the "promotion tournament model," is incapable of optimizing for a society’s well-being if it prioritizes consumption and environmental quality. The effect of tax competition on environmental pollution also differs from area to region, as shown by the heterogeneity study based on the split of Morocco. Tax competition has a strong threshold impact, with opposing direction below and above the threshold, in the center area. Pollutant emissions from vehicles in the East are further exacerbated by the region’s tax rivalry. There is a strong threshold impact of tax competition in the west, and it works in the same manner below and beyond the threshold. As a result, the following five policy recommendations emerge: It is imperative, first, that efforts be made to implement a cross-regional method for controlling pollution. The environmental effects of spilled contaminants tend to cluster in certain areas. Planning environmental governance from a macro perspective is necessary. If we want to improve the state of the environment everywhere, we need to coordinate our efforts as regions. Second, governments at all levels need to devote a growing share of their budgets to environmental preservation. Increased tax competition can improve environmental quality when the amount of government spending on environmental protection is high. This is because it increases both the capacity of environmental governance and the level of public awareness of the need of protecting the environment. While the trend of environmental degradation may be slowed by investing between 1% and 0.5% of national revenue in environmental protection, as shown in industrialized nations. If the percentage is between 2 and 3 percent, then environmental improvements can be made. Third, municipal leaders should hasten the process of modernizing and retooling local industries. Cities should prioritize innovation-driven growth and invest heavily in expanding their knowledge-based agencies and businesses. In addition to fostering tax competition that encourages environmental improvement, the government should increase the pace of producer service development in response to the need for industrial transformation and upgrading. Fourthly, the federal government should give environmental protection accomplishments a greater weight in promotion evaluations and bolster ecological responsibility audits. To accomplish the goal of governments at all levels placing a high value on environmental protection within the official promotion system of the "promotion tournament model," the government should increase the weight of environmental protection achievements in the official promotion assessment and improve the construction of ecological responsibility audit index system. Additionally, providing proper direction to local governments throughout their development planning is facilitated by standardizing the administrative environmental protection system. Finally, the federal government should standardize environmental monitoring and provide administrative guidelines for the environmental protection conduct of local governments. The federal government should strongly encourage state and local governments to shoulder the bulk of environmental protection responsibilities. As a result, local governments are more likely to take measures to safeguard the environment, to grow the local economy in a sustainable way, and to optimize social welfare.
